The article "Application Based on Artificial Intelligence in Substation Operation and Maintenance Management" was retracted in 2023. Reasons: unreliable results or conclusions; concerns about the data; concerns about the results or conclusions; concerns about the peer review.

# Application Based on Artificial Intelligence in Substation Operation and Maintenance Management

**DOI:** 10.1155/2022/7509532

**Published:** 2022-09-01

**Authors:** Xin Zheng, Haihua Zhang, Junyi Shi

**Affiliations:** State Grid Jiangsu Electric Power Co., Ltd, Extra-High Voltage Branch Company, Nanjing 211102, China

## Abstract

To fulfill state grid Industry's demands for smart and digitized business growth, traditional technological approaches have fallen short. Artificial intelligence (AI) technology enables coming up with solutions because electricity business types and volumes are constantly expanding and developing. Intelligent automation was a part of China's smart grid development from the outset, and it continues to grow in the country's electricity system. Smart substation operations and maintenance could benefit from the use of this system. There are new technological tools and theoretical concepts for the repair and control of power equipment owing to AI's advancements in performance, accuracy, and self-learning capacity in the detection, forecasting, improvement, and judgment jobs. Substation operations and maintenance management are examined in this research using a new hybridized convolutional neural network and tweaked long short-term memory (HCNN-TLSTM) technique. Normalization is used to gather and preprocess the data immediately. Kernel-based linear discriminant analysis (K-LDA) is used to extract the features. A substation's functioning and maintenance can then be investigated using the new approach. The genetic algorithm (GA) is used to improve the effectiveness of the proposed method. Finally, the presented technique's performance is analyzed and compared with specific current models to achieve the largest performance in the proposed method for the management of substation operation and upkeep.

## 1. Introduction

Tibet was chosen after the state grid narrowed its search to 5 typical environments throughout the country for the construction of five composite insulating material aging stations. Higher elevation and more UV rays are at Inner Mongolia's Yangbajing. Genhe is cold, while Xinjiang, Turpan, and Henan are hot. Together, the five-building sites in “Zhengzhou” (climate of the Central Plains) and Fujian Meizhou Island (salt fog of the marine) make up an ageing testing platform for composite materials that covers diverse typical climatic and environmental features. The Genhe Aging Test Station is built, operated, and maintained by the State Grid Mengdong Electric Power Research Institute (Wang et al. [1]).

Compliance with technical specifications for building smart laboratories and substations, as well as responses to requirements for building an IoT system, will be required. The “Genhe Extreme Cold Aging Test Station” in Inner Mongolia will be used for this, and a remote monitoring platform in Hohhot will be established utilizing current technologies. It is possible to remotely monitor the progress of test products by using a combination of on-site implementation of various sensors in the surrounding environment, advancement, and troubleshooting of different sensors APPs, mobilization, arrangement of local meteorological monitoring, and so on. Putting it into action is the key to success. So that the test station's operation and maintenance staff may always keep an eye on the test results, deploy different sensors from the primary equipment monitoring system on-site and build and debug various sensor APPs to enable remote controls of the test performed through clever controller (Wan et al. [2]). The correct response to crises at the station.

Maintaining and eliminating faulty substations is currently the primary responsibility of the local smart substation maintenance department. Because of the distinctions between smart substation administration and traditional substation administration, Figure 1 depicts the six primary procedures used to carry out smart substation maintenance.

AI technology may be used to improve the degree of intelligent and intensive grid operation and maintenance, as well as to promote the comprehensive operation and maintenance of transmission and transformation equipment status, in this context, as well. Among the most crucial technological tools for progressing in a targeted and effective manner, domestic intelligent substation maintenance is in charge of substation upkeep and removal at the current count. An intelligent substation maintenance management system is needed because of a lack of a clear distinction between intelligent and conventional substation methods. Checking and assessing the status of electrical substation equipment is made possible by the acquisition of relevant data. Asset condition and risk evaluation are the two most important components of automated substation maintenance works (Song et al. [3]). Accurate evaluation of power equipment status affects substation risk assessment and maintenance. It is crucial for state-maintained smart substations. Scientific methodologies must be utilized to analyze substation equipment and formulate maintenance policies. Develop substation maintenance strategy based on risk assessment. The state's most important maintenance plan is for substation equipment. Substation equipment should be overhauled on schedule according to a company-wide strategy. The maintenance plan implementation involves three phases: planning, execution, and summary. Assess substation maintenance. Evaluating substation equipment overhaul efficacy tests the plan's execution. Work reports must be completed by operations personnel once the overhaul plan has been implemented and they have verified that all equipment is in good working order with the person in charge of the overhaul work. The control center receives updates from the operational crew on the results of the overhaul. Human cognition may be replicated and expanded via artificial intelligence. By using robots that are capable of learning and reasoning, it is hoped to eventually replace humans with machines. It is possible to use AI data analysis technologies, like expert systems and uncertainty reasoning as well as machine learning and intelligent optimum computations. Physical signals, photographs, videos, texts, audio, and other integration of data are all examples of data streams for transmitting power and conversion equipment, repair, and maintenance (Yang and Yao [4]).

Multimodal machine learning analyses data from several modalities. Multimodal learning uses machine learning to interpret and comprehend multisource modal information. Multimodal machine learning combines data for improved feature representation, extraction, and identification. The multimodal learning model integrates and learns multisource information from the model mechanism, not only splicing separate models and turning on their respective “switches” in different contexts. Multimodal learning minimizes duplication across modalities complementarily, which improves learning. Multimodal transfer learning is common. State Grid's “Three Collections and Five Majors” have all been unattended smart substations. Independent operation and maintenance produce additional contradictions. Considering human resource utilization efficiency, time cost, transit cost, and the constant reduction of operational people under large-scale operation and maintenance, smart substations may increase operation and maintenance efficiency (Wang et al. [5]). Due to AI's improvements in performance, accuracy, and the ability to learn on its own in jobs like detecting, forecasting, improving, and judging, there are now new tools and ideas for fixing and controlling power equipment.

The remainder of the description is divided into five parts: part 2: related works and problem definition, part 3: the proposed works used, part 4: result and discussion, and part 5: conclusion.

## 2. Related Works

Kitak et al. [6] demonstrate that the transmission substation's reliability-centered maintenance (RCM) is the subject of this study. An optimization algorithm was used to design and carry out the maintenance procedure. The dependability of the power system functioning, maintenance costs, and related hazards were all taken into consideration in this maintenance approach. For the first time, all maintenance activities are treated as part of the preprocessing and optimization process for reliability-centered maintenance, making the paper unique. Yan et al. [7] introduce integrated automation system of high-speed rail traction substations has limited operational data, low intelligence, and poor identification accuracy. To address these issues, a novel technique of intelligent operation and maintenance has been presented. Zou et al. [8] examine power robots in domestic and international research and their structural characteristics and functions are analyzed for a variety of power applications, including overhead line inspection, substation inspection, live working of distribution lines, and cable channel power equipment inspection and maintenance. Ivanković et al. [9] discuss the existing approach to maintenance management at hops, Croatia's only transmission system operator, as well as potential enhancements to equipment maintenance efficiency via the use of supervisory control and data acquisition (SCADA) data. Zhang et al. [10] focused on the substation project costs thorough cost calculation methods to help a power grid operator better control the cost of constructing a new substation. Sun et al. [11] thoroughly evaluate and contrast the vector model graphics platform in terms of analyzing performance, visual impact, operational effectiveness, reliability, memory size, and expandability. Additionally, three areas of power equipment operation evaluation, maintenance training, and asset management are used to highlight the application of vector model data in substation operation and maintenance. Li and Liu [12] introduce the method of remote intelligent management platform, which uses current mobile Internet and artificial intelligence to realize the “Internet of Everything” and human contact at all stations under the law, to make it an intelligent service system with thorough state awareness, effective data handling, and simple and adaptive implementation. Zhang et al. [13] describe the power system's automation and intelligence level has significantly increased owing to the use of artificial intelligence technologies, which has also accelerated the smart modernization of the power sector. The implementation models, fundamental assumptions, and potential uses of artificial intelligence technology in the power system will serve as the starting points for the subsequent discussion. Zhang et al. [14] illustrate the concept of an artificially intelligent power system that is used. It initially provides a thorough analysis of the concept before outlining how operation and maintenance have evolved inside the Chinese power system. In addition, many generic technologies—including protection systems, crucial operation, particularly based on deep learning—as well as various approaches used in the substation, converter station, and new energy are addressed. Bai et al. [15] offer the whole chain of operations from model creation to application development, covering sample analysis, model construction, and common distribution; they present a power system AI platform design and implementation plan. Salihu and Zayyanu [16] examined the samples taken from vegetable farms in Zamfara State, Nigeria, for thermodynamic and organophosphate agrochemicals. It was utilized to assess the testing method and the produced data using QuEChERS with GC-MS. Wang et al. [17] proposed 5G communication system architecture that is used in this study to implement wireless heterogeneous networking. A three-dimensional registering approach that relies on ORB-Tanimoto has been presented in light of the possibility of considerable time delays and inaccuracies in the three-dimensional enrollment process of augmented reality technology and the necessity for security and real-time efficiency in substation operations. First, the Tanimoto is used to integrate ORB recognition with the three-dimensional registering approach for correlating characteristics. Luo et al. [18] examine the use of intelligent technologies in traditional substations, such as patrol robots, manipulating robots, artificial intelligence (AI), augmented reality (AR), online monitoring, and so forth. Zhaoli et al.'s [19] goal was to enhance the operational stability of the substation DC system and achieve lean operation and maintenance; this study provides a design scheme for the DC power management system after considering the current and new DC power management issues. Wang et al. [20] focused on the substation's functioning, as well as the causes and effects of the station's energy consumption. Substation equipment is briefly described in terms of its energy-related functions, classifications, and uses. Based on an examination of the energy consumption data collecting technique, calculation foundation, and analysis method, the monitoring application of power equipment in the substation is developed. The findings of energy monitoring at the substation are discussed.

### 2.1. Problem Statement

A power transformer's insulating effectiveness may be damaged by a combination of multiple variables including loaded conditions, excessive heat, residual vibration, operational circumstances, and the meteorological environment. It is important to note that all of the information gathered throughout this technique gives details on equipment functioning conditions and problem propagation across the process. These platforms, which include production planning systems, smart metering, geospatial and weather patterns systems, and other types of power network implementation, have identified a wide range of different distinctions in data relating to the ability to operate state of the power distribution transformer. Improved diagnostic assessment and forecast results may provide a more reliable point of reference for equipment decision-making optimization, enhancing converter declarative programming still further.

## 3. Proposed Work

To guarantee the security of the substation's hardware and surroundings, initially, physical labor was used to check substation hardware. Nevertheless, as the development of large power networks progresses, the frequency of substations continues to rise. So, in this part, the proposed HCNN-TLSTM technique is employed to predict the power equipment' illustrated as depicted in Figure 2.

### 3.1. Dataset

Under this research, we make use of a relatively large electric grid database (Lyu et al. [21]), which includes (1) profiles of power users, including geographical data, login details, and user types; (2) profiles of electricity substations; and (3) time-series data on user power usage. Between March 10 and April 13 of the year, researchers in Xinjiang Province obtained the information.

### 3.2. Data Preprocessing

The long-term accumulation of test/patrol examination data, malfunction records, and servicing documentation are what make up the bulk of the textual data for power transformers. The state's regular maintenance will be guided by the information provided in this report. Investigation on the assessment of power equipment breakdown through trouble tickets has already been done by foreign countries; however, because of the clear distinctions in part-of-speech and grammar structure between Chinese and English text, it is critical to creating important information for the features of power Chinese text analysis. China's text categorization difficulty is broken down into a series of five steps of processing.

#### 3.2.1. Stop Word Removal

The field of computer science known as “natural language processing” (NLP) is more particularly the field of “artificial intelligence” (AI) that is focused on providing machines the capacity to comprehend written verbal speech like that of humans. An important NLP preprocessing step has been employed in many different contexts. It is only a matter of eliminating words that appear in a large number of different documents throughout the corpus. Stop words, such as articles and pronouns, are what they are called. Eliminating certain stop words as the very first step in pretreatment has shown to be quite significant.

#### 3.2.2. Stemming

As the name suggests, stemming is the act of resolving words to their root word stem, which is referred to as a lemma. Like an attribute selection strategy, text analysis technologies frequently make use of this procedure.

#### 3.2.3. Document Indexing

By removing certain phrases from the generated document, indexing can be made more efficient, which is why document indexing is so important. Document indexing is the process of selecting the right collection of keywords from the entire corpus of documents and giving weights to such keywords for every individual text, thereby converting all files into a vector of keyword weights. The number of times a term appears in a document, as well as the total number of times it appears, determines the weight assigned to it.

#### 3.2.4. Term Weighting

Term weighting is critical to the categorization system's accomplishment. Because distinct terms in a text have varying degrees of value, the term weight has been used to indicate the significance of each term.

#### 3.2.5. Dimensionality Reduction

Text mining algorithms can handle data with fewer terms thanks to dimension reduction, which reduces the dimensions used by clustering approaches. It is possible to shrink a vector's size by using a method known as singular value decomposition.

The input dataset is isolated from the training and testing datasets. In the training dataset, there is a variable that must be expected or identified as an output. The patterns uncovered in the training dataset are applied to the test dataset by all prediction and classification algorithms.

### 3.3. Feature Extraction Using K-LDA

Feature extraction employs kernel-based linear discriminant analysis (K-LDA). To eliminate the curse of dimensionality, save resources, and minimize dimensional expenses, K-LDA projects characteristics from a higher-dimensional space onto a lower-dimensional space. When within-class frequencies are mismatched and performance is tested using randomly produced test data, K-LDA assures maximal separability by raising the variance to within-class variation ratio in each data. It is used in data detection to solve the classification problem. Our goal is to develop a method that uses LDA rather than Principal Component Analysis to improve accuracy.

Make the test sets and data for categorizing the source field. Data collections and trial matrices are created as needed. Let us express the data sources as a data matrix using the following format to make things easy to understand.

(1) $$\begin{array}{c} \text{Set }1=\left[\begin{array}{cc} \begin{array}{c} b_{11}\\ b_{21}\\ \begin{array}{c} ..\\ ..\\ b_{n1} \end{array} \end{array} & \begin{array}{c} b_{12}\\ b_{22}\\ \begin{array}{c} ..\\ ..\\ b_{n2} \end{array} \end{array} \end{array}\right],\\ \text{Set }2=\left[\begin{array}{c} \begin{array}{c} c_{11}\\ c_{21}\\ \begin{array}{c} ..\\ ..\\ c_{n1} \end{array} \end{array}\\ \begin{array}{c} c_{12}\\ c_{22}\\ \begin{array}{c} ..\\ ..\\ c_{n2} \end{array} \end{array} \end{array}\right]. \end{array}$$

Calculate the overall mean as well as the mean of each data collection. Let *g*_1_ be the means of sets 1 and 2 and *g*_2_ be the mean of the total data obtained by combining the two sets. The average of both the complete data acquired by combining sets two and three is given in the following equation.

(2) $$\begin{array}{c} \pi_{3}=g_{1}\times \pi_{1}+g_{2}\times \pi_{2}, \end{array}$$

Here are the classes' a priori probabilities. The probability factor is considered to be 0.5 in this basic two-class situation.

K-LDA uses both within-class and between-class dispersion to determine class separability requirements. The predicted covariance of each of the classes is the within-class dispersion. Equations (2) and (3) are used to calculate the scatter measurements.

(3) $$\begin{array}{c} R_{u}=\underset{i}{\sum }g_{i}\times \left({\text{cov}}_{i}\right),\\ R_{u}=0.5\times {\text{cov}}_{1}+0.5\times {\text{cov}}_{2},\\ {\text{cov}}_{i}=\left(y_{i}-\pi_{i}\right){\left(y_{i}-\pi_{i}\right)}^{D,}\\ R_{c}=\underset{i}{\sum }\left(\pi_{i}-\pi_{3}\right)\times {\left(\pi_{i}-\pi_{3}\right)}^{D}. \end{array}$$

The autocorrelation arrays are all homogeneous matrices. Equation (6) is used to calculate the covariance matrix.

This is the variance of a set of datasets, and the elements are the median vectors of each group. As previously stated, the best requirements in LDA are the fraction of some place between scattering inside each scatter. The axis of the modified space is defined by the solution obtained by the maximization of these criteria. On the other hand, the class-dependent transform is employed to choose the optimum criterion. If the LDA is merely a type of category, each type will require its own set of optimizing criteria. For a class-dependent type, the optimal factors are as follows:

(4) $$\begin{array}{c} {\text{criterion}}_{i}=\text{inv}\left(cov_{i}\right)\times R_{c},\\ \text{criterion}=\text{inv}\left(R_{u}\right)\times R_{c}. \end{array}$$

Every L-class issue would have L-1 nonzero eigenvalues. This is due to equation (9)'s limitations on the groups' median indices. The anti-eigenvalue vectors are utilized to specify the transformation. In our two-class example, they show the direction of the primary eigenvector, which provides the most discriminating information. After collecting the transformation matrices, we convert the metrics using either a single LDA change or a classifier change, depending on the conditions. As seen in the images, converting the entire range of data to only one vector provides indicated boundaries for classifying data. The choice zone in transformed space is a straight line that divides the converted data sources. When it comes to LDAs that are dependent on a class,

(5) $$\begin{array}{c} {\text{transformed}}_{{\text{set}}_{\_i}}=\text{transform}\_i^{D}\times \text{set}\_i,\\ {\text{transformed}}_{{\text{set}}_{\_i}}=\text{transform}\_{\text{spec}}^{D}\times \text{data}\_{\text{set}}^{D}. \end{array}$$

Similarly, the test vectors are transformed and categorized using the calculation between each class means and the test vectors. These examples show how to use K-LDA classification to classify a two-class situation. The original data sets are shown, as well as the identical data sets following modification. These examples show how transformation limits the accuracy of categorization. Although the classes in this example were properly established, in instances where classes overlap, finding a selection area in the image space may be challenging, necessitating conversion. The axis with the biggest eigenvector yields the optimal transformation. These are particularly fascinating because they demonstrate how quadratic development may be understood as putting data into the eigenvectors' highest discerning planes.

### 3.4. AI-Based Data Analysis Using the HCNN-TLSTM Technique

#### 3.4.1. Convolutional Neural Network (CNN)

CNN retrieves features from the input data and generates a dense and complete feature vector from the source data using local connections with weight sharing. Data features were retrieved using CNN for this inquiry. The CNN includes the source, convolutional layer, pooling layer, fully connected layer, and destination.

#### 3.4.2. Tweaked Long Short-Term Memory (TLSTM)

We apply the TLSTM approach in the prediction phase for effective prediction. This method can be applied in all states for the best results. The recurrent neural network (RNN) succeeds in comprehending time-series data due to its internal state's ability to reflect dynamic temporal properties. Gradient fading is caused by gradually multiplying the weight matrix and the reciprocal of the tanh (from 0 to 1) function, which increases as the data interval (the indicated fixed length) grows longer. As an extended type of RNN, LSTM can successfully decrease gradient fading in standard RNN. The LSTM uses a gate control technique to determine whether an input should be recalled or rejected, and it can use long-time sequence data to some extent. The LSTM framework is shown in Figure 3.

To replace RNN neurons, LSTM employs memory blocks with three types of gates (input, forget, and output gates). Equations could be used to express the data calculated inside LSTM memory blocks [3–8].

(6) $$\begin{array}{c} e_{t}^{g}=\sigma \left(B^{g}X_{t}+R^{g}h_{t-1}+\xi^{g}\right),\\ e_{t}^{k}=\sigma \left(B^{k}X_{t}+R^{k}h_{t-1}+\xi^{k}\right),\\ m_{t}^{c}=\text{tanh}\left(B^{m}X_{t}+R^{m}h_{t-1}+\xi^{m}\right),\\ c_{t}=e_{t}^{g}*c_{t-1}+e_{t}^{k}*m_{t}^{c},\\ e_{t}^{o}=\sigma \left(B^{o}X_{t}+R^{o}h_{t-1}+\xi^{o}\right),\\ c_{t}=e_{t}^{o}*\;\tanh\left(c_{t}\right), \end{array}$$

Here, *e*_*t*_^*g*^ = forget gate during the time (t), *e*_*t*_^*k*^ = input gate during *t*, *e*_*t*_^*o*^ = output gate during *t*, *m*_*t*_^*c*^ = candidates of input to be stored at *t*, *c*_*t*_ = memory cells at *t*, *h*_t_ = hidden state at *t*, *X*_t_ = input vectors at *t*, *ξ*^*g*^ = bias vector of forget gate, *ξ*^*k*^ = bias vector of input gate, *ξ*^*o*^ = bias vector of output gate, and *ξ*^*m*^ = bias vector of candidates of the input. Then, *B*^*g*^, *B*^*k*^, *B*^*m*^, *B*^*o*^, *R*^*g*^, *R*^*k*^, *R*^*m*^, and *R*^*o*^ are related weight matrices. The “Hadamard product” was indicated as *∗* among two matrices. Furthermore, *σ* and tanh were termed activation functions.

The projected judgments in some regression scenarios are influenced not only by the original inputs but also by subsequent inputs. By combining the original and subsequent inputs, TLSTM can enhance prediction accuracy. Forward long short-term memory and backward long short-term memory are the two types of TLSTM. The results of both forward and backward computations, whose designs are congruent with the architecture of LSTM memory blocks, make up TLSTM's final output.

#### 3.4.3. Genetic Algorithm (GA)

The genetic algorithm, which is based on natural selection, the mechanism that promotes biological evolution, is a technique for resolving both limited and uncontrolled optimization issues. A population of unique solutions is repeatedly modified by the genetic algorithm. The conventional algorithm includes encoding, initialization, choosing, crossover, mutation, decoding, and other basic GA activities. The use of the GA improves searching and optimization in such operations. Programming is the initial step. The survival of the fittest principle states that evolution will produce ever-better approximate results after the first generation of a population. Physical fitness is used to select individuals for future generations. Natural genetics can be utilized to create a new group that is similar to the original one through crossover and mutation. The GA process flow diagram is shown in Figure 4.

 The most significant part of the forecasting approach is HCNN-TLSTM. A convolutional layer, a pooling layer, and a flattening layer make up the CNN system. For the Conv2d layer, it has been allocated to the *m*-layer. By adjusting the volume of the CNN convolution kernel, it is possible to extract features from datasets from multiple periods. To optimize current information, the size of the convolution kernel is set at [*n* × *n*]. When computing the set of genes to employ, the GA also displays the proportion of convolution kernels within each convolutional layer. The *m*-layer pooling layer (Maxpooling-2D) is also tuned to *m*-layer and has a size of [*n* × *n*]. Batch normalization is added before the pooling layer as a performance gain. The data is then flattened to retrieve global features from compressed data. The data is fed into the TLSTM unit to create a forecast.

The addition of TLSTM system components improves the model's ability to anticipate future events, according to studies. As a result, the GA's specific genes are set to the relevant number of neurons in each TLSTM layer, and the *x*-layer TLSTM module is picked. Dropout is a TLSTM feature that prevents problems with fitting. Finally, Dense creates a vector in the format specified, which is subsequently used in forecasting.

The genetic algorithm-based HCNN-TLSTM approach proposed in this research is an improvement on the HCNN-TLSTM algorithm. The HCNN-TLSTM method has been proved to be useful in numerous experiments, particularly when making predictions. The genetic algorithm-based HCNN-TLSTM approach computes data produced from a convolutional neural network as a feed to LSTM to forecast time-series data. During long-term time-series forecasting, TLSTM will prevent gradient vanishing. Many studies use time-consuming and labor-intensive manual selection procedures like grid search to find parameters for the HCNN-TLSTM model, making it difficult to find the most optimal parameters. As a result, this paper chooses a genetic algorithm and employs the genetic and mutation phase of the algorithm for scientific parameter estimate, which is more effective than previous methods.

A TLSTM is made up of many convolution kernels and neurons, with the number of convolution kernels and neurons changing. When the criterion or requirements are met, the most appropriate individual is chosen, and their genes are employed as variables in the HCNN-TLSTM.

Here is how each group's fitness function (*F*) looks:

(7) $$\begin{array}{c} F=\frac{1}{e}\left(1+u\left(1-\frac{M_{c}}{M_{t}}\right)+v\left(1-\frac{M_{\text{TLSTM}}}{M_{t}}\right)\right). \end{array}$$

Here, *e* = error (Mean Absolute Percentage Error (MAPE) is used as an “*e*”), *u* = convolution layer's impact on system quality, *v* = TLSTM's impact on system quality, *M*_*c*_ = quantity of convolutional kernels, *M*_TLSTM_ = quantity of LSTM's neurons, and *M*_*t*_ = summation of *M*_*c*_ and *M*_TLSTM_.

The fitness “*F*” of GA-based HCNN-individual TLSTM and MAPE (“mean absolute percentage error”) was also created as an inverse relationship; thus, the MAPE is used to determine individual fitness, allowing for an evaluation of the model's effectiveness and the establishment of the final attribute values. When compared to choosing all the variables of the HCNN-TLSTM model with the best performance using an exhaustive technique, this will save a significant amount of time. As shown in Figure 5, our research proposes a thorough modeling approach based on the genetic algorithm-based HCNN-TLSTM framework for producing power equipment breakdown forecasts and evaluating their performance.

## 4. Performance Analysis

In this stage, the suggested technique's performance is evaluated, and a comparison analysis is computed by comparing it to some existing techniques (Text CNN [Chen et al. [22]], CAD-IOMPSE [Song et al. [3]], Glove-BiLSTM-Attention [Chen et al. [23]], and DA-BiLSTM [Li et al. [24]]) for predicting power equipment breakdowns.

The proposed technique is used to anticipate the breakdown of power devices using data from the China power grid. Furthermore, key performance measures of the proposed technique, such as MAPE, precision, recall, veracity, *R*^2^-value, and training time, are studied and compared to existing techniques in a comparative analysis to show that our technique has the best prediction.

The breakdown of power equipment can be characterized as either a good or bad event. We separated the sample into four trials [i.e., “A = true positive,” “B = true negative,” “C = false positive,” and “D = false negative”]. Our method anticipates each piece of data separately, so we arrange them according to their predictions and use the data as examples. Certain indicators are evaluated in this area for our planned study for predicting the breakdown of power equipment. These figures are shown below.

### 4.1. Performance Metrics

#### 4.1.1. MAPE

The average divergence between projected and actual tourist activity at picturesque sites is measured by MAPE. The result of MAPE for both proposed and existing strategies is indicated in Figure 6. This metric is assessed for both strategies by using the below equation. From this investigation, the proposed technique has the lowest MAPE (19.13%) compared with existing techniques.

(8) $$\begin{array}{c} \text{MAPE}=\frac{1}{n}\overset{n}{\underset{i=1}{\sum }}\left|\frac{W_{i}-P_{i}}{W_{i}}\right|. \end{array}$$

Here, *m* = summation of samples, *W*_t_ = real value, and *P*_t_ = predicted value.

#### 4.1.2. Precision

It is a measure of how many power equipment breakdown predictions are accurate. This determines how precise our results are when comparing to other conventional results. The result of precision for both proposed and existing strategies is indicated in Figure 7. Equation (20) is used to assess the precision for both training and testing datasets in proposed and existing techniques and also this metric is indicated in percentage. Here, the proposed technique attains the highest precision rate in the proposed technique's training set (93.58%) than the testing set (88.21%). Moreover, the precision rate of both the training and testing datasets has the highest effectiveness than that of existing techniques.

(9) $$\begin{array}{c} \text{precision}=\frac{A}{\left(A+C\right)}. \end{array}$$

#### 4.1.3. Recall

It is a calculation that indicates how many right positive predictions were produced out of the total number of possible positive predictions. In contrast to accuracy, which only comments on positive predictions that are correct, recall acts as an indicator of correctly predicted that is incorrect. The result of recall for both proposed and existing strategies is indicated in Figure 8. Equation (21) is used to evaluate the recall rate of proposed and current approaches for both training and testing datasets, and this measure is expressed in percentage. The proposed technique achieves a higher recall rate in the training set (94.41%) than in the testing set (87.20%). Furthermore, both the training and testing datasets have the best recall rate compared to previous approaches.

(10) $$\begin{array}{c} \text{Recall}=\frac{A}{\left(A+D\right)}. \end{array}$$

#### 4.1.4. *R*^2^ Value

The predicted models' anticipated *R*-squared reveals how accurate it is at predicting fresh measurements' reactions. The result of *R*^2^ for both proposed and existing strategies is indicated in Figure 9. For both training and testing datasets, this metric is used to evaluate the accurateness of the new measurements' reactions to proposed and present techniques, and this metric is expressed in percentage. In the training set (98.71%), the proposed technique obtains a greater precision rate than in the testing set (91.52%). Furthermore, when compared to earlier techniques, both the training and testing datasets had the highest *R*^2^ rate.

#### 4.1.5. Veracity

Veracity is the proportion to which information is exact, accurate, and dependable. The result of veracity for both proposed and existing strategies is indicated in Figure 10. In this investigation, this metric is used to evaluate the conformity of proposed and current approaches for both training and testing datasets, and this measure is represented in percentage. The proposed technique achieves a higher veracity rate in the training set (96.9%) than in the testing set (89.12%). Furthermore, both the training and testing datasets had the most excellent veracity rate when compared to previous approaches.

Figure 11 shows the training time of proposed and current power equipment breakdown predicting techniques. Compared to current methods, ours takes 250 seconds in training. Based on this research, conventional methods achieve maximum training time whereas our method achieves minimum training time.

Compared with existing approaches, precision, recall, and veracity of the proposed algorithm are very high and effective. Initially, when several trials yield the same outcome with little variation, precision is necessary. Hence, precision is effective and plays a vital role in comparison. Second, recall is the percentage of pertinent instances that were found. It gives accurate results. Veracity is being used to know how the system is implemented in real time and how it is beneficial. So, it is being voracious or needy in quality or state.

## 5. Discussion

In this part, the comparative analyses of the metrics in both proposed and existing techniques are illustrated. It is possible to forecast the state of an item of equipment by monitoring and evaluating its status. From the equipment's historical and real-time data and the grid's operational and environmental data, indicators or the shifting pattern of important factors that can anticipate its future operation more accurately can be identified. The forecast of the present condition of power distribution and transformation apparatus is typically based on some leading factors as the forecasting objective due to the complicated working conditions and various index factors. In this investigation regarding the substation power equipment breakdown forecasting, the various performance metrics are estimated for both proposed and current techniques as depicted in Figures 6–10. The current techniques have inconsistent efficiencies due to their certain shortcomings. For accuracy and *F*_1_ scores, Text CNN produced better results in (Chen et al. [22]). However, no additional measures are calculated, resulting in a reduction in prediction effectiveness. The CAD-IOMPSE approach also generates superior accuracy, recall, and *F*-measure results (Song et al. [3]). However, the error metric is not given, which leads to inefficient results. Chen et al. [23] proposed GloVe-BiLSTM-Attention-based defect textual classification method, which has been tested for precision, recall, and *F*_1_-score. DA-BiLSTM framework on basic power grid fault texts was applied to reduce misclassifications caused by data interruption (Li et al. [24]). According to the results of Chen et al. [23] and Li et al. [24], the rate of certain measures was improved, but certain metrics were not determined, which reduced the prediction's performance. Finally, we accomplish the greatest degree of veracity, precision, recall, and *R*^2^, as well as the lowest rate in MAPE and training time by employing the proposed method than those existing methods.

## 6. Conclusion

There has been a spike in the volume of power grid hardware resources, and also a rise in the number of data was needed to maintain the operation and maintenance of these systems. When it comes to activities such as detection, forecasting, improvement, and judgment, the latest innovative methods and research topics for power equipment maintenance and operation are being provided by AI technological innovation and breakthroughs in effectiveness, reliability, and self-learning capability. While the standard cost calculation system for operating and maintaining power grid equipment does not strictly fall under the scope of industry standards, it is based on the standard operating database that is currently in use, actual operating data, and field investigations, and it integrates different substation business activities. This paper suggested a new HCNN-TLSTM technique to manage such operations and maintenance issues of the powerful hardware assets in the substation. Here, also the breakdown of the power equipment was forecasted by employing the suggested technique. Chinese text analytics was accomplished using various methodologies, such as stop word removal, stemming, document indexing, and dimension reduction. K-LDA technique was utilized to retrieve the significant characteristics from the normalized text data. Followed by, the proposed technique was applied to predict the power equipment's breakdown risks. At last, the proposed technique was carried out in the comparative analysis with certain existing techniques to attain the greatest effectiveness in the operation and maintenance of the powerful hardware assets in the power substation in terms of veracity, precision, recall, and MAPE, training time, and *R*^2^-value. Quality of the data, data hurdles, and a dearth of atypical samples are all impeding the development of applications for AI technology in these contexts. It is imperative that in the future we concentrate on enhancing the management and monitoring of data records and investigating better and more sophisticated analysis techniques to encourage the cognitive growth of hardware condition management even further.

## Figures and Tables

**Figure 1:** Primary procedures for smart substation maintenance.

**Figure 2:** Complete procedure of this research.

**Figure 3:** Framework of typical LSTM.

**Figure 4:** Procedure of GA.

**Figure 5:** Framework of prediction using genetic algorithm-based HCNN-TLSTM.

**Figure 6:** MAPE outcome.

**Figure 7:** Precision outcome.

**Figure 8:** Recall outcome.

**Figure 9:** *R* ^2^ outcome.

**Figure 10:** Veracity outcome.

**Figure 11:** Training time.

## Data Availability

The data used to support the findings of this study are available from the corresponding author upon request.
